This article has been retracted.

# Gastric Volvulus: A Rare Etiology of Acute Chest Pain

**DOI:** 10.7759/cureus.19067

**Published:** 2021-10-26

**Authors:** Maryam A Sultan, Alhanouf A Hakami, Meshari I Alshabri, Shahad A Alsuwailem, Nuwayyir E Aqeel, Rajis N Aldosari, Tariq H Alrazhi, Khaled A Al-Wesabi, Abdullah A Alzayed, Majed A Alanazi, Aioub S Al Yousef, Ahmed S Alromaihi, Roaa M Aljadeed, Sahar H Alomar, Malak Alshammari

**Affiliations:** 1 College of Medicine, Jazan University, Jizan, SAU; 2 College of Medicine, King Saud University, Riyadh, SAU; 3 College of Medicine, Alfaisal University, Riyadh, SAU; 4 College of Medicine, Imam Mohammad Ibn Saud Islamic University, Riyadh, SAU; 5 General Practice, Dhahran General Hospital, Dhahran, SAU; 6 College of Medicine, Dar Al Uloom University, Riyadh, SAU; 7 College of Medicine, King Saud Bin Abdulaziz University for Health Sciences, Riyadh, SAU; 8 College of Medicine, Jordan University of Science and Technology, Irbid, JOR; 9 College of Medicine, Arabian Gulf University, Manama, BHR; 10 College of Medicine, Imam Abdulrahman Bin Faisal University, Dammam, SAU

**Keywords:** operative laparoscopy, computed tomography (ct ), hematemesis, gastric volvulus, chest pain, case report

## Abstract

Chest pain is one of the most common complaints in the emergency department. The etiologies of chest pain include a wide spectrum of conditions, ranging from mild and self-limited to life-threatening conditions. Gastrointestinal origins of acute chest pain, including esophageal, gastric, and biliary conditions, are not uncommon. We present the case of a 67-year-old man who presented to the emergency department with chest pain of three hours duration with pressure-like quality. The pain was associated with sweating, palpitation, nausea, and vomiting. The past medical history of the patient was remarkable for ischemic heart disease and percutaneous cardiac intervention. Both the electrocardiograph and cardiac biomarkers were normal. The patient experienced severe episodes of vomiting with one episode containing a small amount of blood. Upper gastrointestinal endoscopy revealed distorted anatomy of the stomach. Subsequently, the patient underwent a computed tomography scan which demonstrated an organoaxial gastric volvulus. The patient was resuscitated and underwent laparoscopic repair of the volvulus. Acute gastric volvulus is a very rare etiology of chest pain. Despite its rarity, physicians should keep a high index of suspicion of this condition after excluding the possible cardiac causes of chest pain.

## Introduction

Chest pain is one of the most common complaints in the emergency department. It is estimated that chest pain accounts for over seven million visits to the emergency department annually in the United States [1]. The etiologies of chest pain include a wide spectrum of conditions, ranging from mild and self-limited to life-threatening conditions. The initial evaluation of acute chest pain should include appropriate history, physical examination, electrocardiograph, and cardiac biomarkers in order to exclude the possibility of acute myocardial infarction. However, it should be remembered that less than 15% of patients with acute non-traumatic chest pain have acute coronary syndrome as the cause of their pain [2]. Gastrointestinal origins of acute chest pain, including esophageal, gastric, and biliary conditions, are not uncommon [3]. For instance, gastroesophageal reflux disease is the most common etiology of non-cardiac chest pain [4]. Here, we present the case of an elderly man with a history of ischemic heart disease who presented with sudden central chest pain with similar characteristics of cardiac chest pain. After thorough investigation, the patient was found as having an organoaxial gastric volvulus, which is a very rare clinical entity.

## Case presentation

We present the case of a 67-year-old man who presented to the emergency department with chest pain of three hours duration. He described the pain as pressure-like and was central in a location with no radiation. The pain started suddenly and remained constant. It was associated with sweating, palpitation, nausea, and vomiting. The pain was not relieved by simple analgesia medications. Further, it was exacerbated by exertion. The pain was not related to posture or respiration. He rated the pain as 8 out of 10 in severity. There was no change in urinary or bowel habits. The patient reported no history of anorexia, weight change, or fever.

The past medical history was remarkable for hypertension, diabetes mellitus, dyslipidemia, and stable angina. The patient underwent percutaneous coronary intervention five years ago. He remained symptom-free following the procedure. His medications included captopril 25 mg, metformin 1000 mg, aspirin 75 mg, clopidogrel 75 mg, and atorvastatin 20 mg. He was on regular follow-up visits with the cardiology team with no recent changes in his medications. The past surgical history was remarkable for open appendectomy. He was a retired school teacher. He never consumed alcohol and had a smoking history of 25 pack-years.

Upon examination, the patient appeared sick. He was not in respiratory distress. He was not pale, jaundiced, or cyanosed. His vital signs were a temperature of 36.8℃, pulse rate of 110 bpm, blood pressure of 128/82 mmHg, and respiratory rate of 14 bpm. Cardiac examination revealed a normal S1 and S2 with no added sounds or murmurs. Respiratory examination revealed normal vesicular breathing throughout both lung fields. Abdominal examination revealed a soft and lax abdomen with epigastric tenderness. The electrocardiograph revealed a normal sinus rhythm with normal ST segments. The patient received soluble aspirin, clopidogrel, and sublingual nitroglycerin without clinical improvement. Both troponin-I and creatinine kinase enzymes were not elevated. The other basic laboratory investigation was within the normal limits (Table 1).

**Table 1:** Summary of the results of laboratory findings.

Laboratory investigation	Unit	Result	Reference range
Hemoglobin	g/dL	13.1	13.0–18.0
White blood cell	1000/mL	4.8	4.0–11.0
Platelet	1000/mL	375	140–450
Erythrocyte sedimentation rate	mm/hr	13	0–20
C-reactive protein	mg/dL	5.2	0.3–10.0
Total bilirubin	mg/dL	1.1	0.2–1.2
Albumin	g/dL	3.4	3.4–5.0
Alkaline phosphatase	U/L	50	46–116
Gamma-glutamyltransferase	U/L	48	15–85
Alanine transferase	U/L	60	14–63
Aspartate transferase	U/L	27	15–37
Blood urea nitrogen	mg/dL	17	7–18
Creatinine	mg/dL	1.2	0.7–1.3
Sodium	mEq/L	138	136–145
Potassium	mEq/L	4.5	3.5–5.1
Chloride	mEq/L	106	98–107

The patient experienced severe nausea with an episode of vomiting that contained a small amount of blood. Intravenous omeprazole was administered and resulted in improvement of his symptoms. Then, the patient was prepared for emergency upper gastrointestinal endoscopy which revealed distorted anatomy of the stomach with no gross lesions. Further, the endoscopist could not pass through the pyloric canal. Subsequently, an abdominal computed tomography scan with oral contrast. The scan demonstrated thoracic herniation of the stomach with rotation about its long axis. The lesser curvature was inferior to the greater curvature. Such findings conferred the diagnosis of organoaxial gastric volvulus (Figures 1, 2).

**Figure 1:** Axial CT image. Selected computed tomography image of the chest in the axial plane demonstrating the contrast-filled stomach (arrow) herniated in the thoracic cavity.

**Figure 2:** Coronal CT image. Selected computed tomography image of the upper abdomen in the coronal plane demonstrating the contrast-filled stomach (arrow) rotated along its vertical axis, conferring the diagnosis of organoaxial gastric volvulus.

The patient was resuscitated with intravenous fluid and electrolyte therapy. Nasogastric tube decompression was performed. The decompression of the stomach resulted in reliving the patient’s symptoms. The patient remained symptom-free and was hemodynamically stable. Two days later, the patient underwent laparoscopic surgery for the definitive treatment of the volvulus. The herniated stomach was reduced. Careful examination of the stomach showed no areas of ischemia. The stomach was detorted and gastropexy was performed. The patient tolerated the procedure with no complications. The total operative time was 150 minutes and the estimated blood loss was 50 mL. The patient had an uneventful recovery. He was discharged on the sixth postoperative day. He was followed up for one year and had no active issues.

## Discussion

We presented the case of a 67-year-old man with gastric volvulus who presented with central crushing chest pain with normal electrocardiograph and cardiac biomarkers findings. Gastric volvulus is defined as the rotation of the stomach along its vertical or horizontal axis, which may result in a gastric outlet obstruction of variable degrees with potential ischemia, strangulation, perforation, and sepsis [5]. Early diagnosis of gastric volvulus is of paramount importance as it can lead to a substantial mortality risk if it was not recognized and managed appropriately [6].

As in the present case, gastric volvulus often develops after the fifth decade. Other risk factors associated with the development of gastric volvulus include diaphragmatic eventration, kyphoscoliosis, paraesophageal hernia, hiatal hernia, or phrenic nerve palsy [5]. In the current case, the patient was not known to have a prior history of gastroesophageal reflux disease. Gastric volvulus can be primary or secondary. In the primary form, the volvulus develops due to abnormalities in the gastric ligaments that may result from malignancy, adhesions, or kyphoscoliosis. However, gastric volvulus is more commonly secondary to other anatomic abnormalities like esophageal hernia [7].

The clinical manifestation of gastric volvulus may include acute or chronic presentations. It may present with abdominal pain or chest pain. Further, as in the present case, hematemesis may develop due to mucosal tears resulting from the severe vomiting episodes [5]. It is reported that up to 70% of patients with gastric volvulus present with the triad of pain, vomiting, and inability to pass the nasogastric tube, which is referred to as Borchardt’s triad [6]. However, considering its rarity, gastric volvulus is not considered as the underlying etiology of such symptoms. The initial laboratory investigation could suggest evidence of volume depletion and electrolyte disturbances.

The definitive treatment of gastric volvulus is immediate or delayed surgical management. The surgery can be delayed in case the nasogastric decompression was not successful [8]. In the present case, the laparoscopic approach was performed as the patient was hemodynamically stable with no metabolic derangements.

## Conclusions

Acute gastric volvulus is a very rare etiology of chest pain. Despite its rarity, physicians should keep a high index of suspicion of this condition after excluding the possible cardiac causes of chest pain. A computed tomography scan can make the diagnosis accurately. Laparoscopic treatment is a feasible and safe option for the management of acute gastric volvulus.
